The article "Building and Realizing the Obstetrics and Gynecology Nursing Management Platform by Computer Information Technology under the Concept of Mindfulness Intervention" was retracted in 2023. Reasons: suspected computer-generated content; unreliable results or conclusions; lack of ethics approval or compliance; missing or withdrawn patient consent.

# Building and Realizing the Obstetrics and Gynecology Nursing Management Platform by Computer Information Technology under the Concept of Mindfulness Intervention

**DOI:** 10.1155/2022/6297934

**Published:** 2022-03-21

**Authors:** Lijuan Huang, Xianmei Cui

**Affiliations:** ^1^Shanxi Medical University, Shanxi, China; ^2^Network Education College of Shanghai Jiaotong University, Shanghai, China

## Abstract

Nursing management of the gynecology department is one of the challenging issues and needed to be resolved through effective utilization of the available technology. In this paper, we are going to address this issue and try to establish an obstetrics and gynecology nursing management platform used to monitor and evaluate the mental health of pregnant women. Firstly, computer information technology is adopted, and the obstetrics and gynecology nursing management system is established. Secondly, after adopting the system to intervene in the mental state of patients with mindfulness, the system timely monitors the pregnant women's physical health indicators and mental health level data. With the help of the computer data analysis system, the obstetrics and gynecology management platform is built to carry out timely mindfulness interventions for pregnant women. The established system can reach high accuracy in identifying negative emotions of pregnant women, and the accuracy can reach 89.7%. It shows that the established system can timely and accurately intervene and regulate the pregnant woman's bad psychological state, effectively improve the pregnant woman's sleep quality during pregnancy, and enhance the pregnant woman's sleep effect. The effectiveness and feasibility of Internet mindfulness interventions for improving sleep quality during pregnancy has been confirmed. This has important practical significance for the digital and intelligent development of the medical care management platform.

## 1. Introduction

Pregnancy [1–3] is a strong stress response for women. During pregnancy, women not only face a series of physiological changes, but due to increased economic pressure and changes in social roles, women may also experience a series of changes in their psychological state. Under extremely strong psychological pressure, the frequent fluctuations of a woman's emotions can even cause health problems in varying degrees. Relevant studies have shown that 82% of pregnant women have sleep quality problems during pregnancy, manifested as difficulty in falling asleep, insomnia, and an increased number of night awakenings. Sleep problems and negative emotions will not only affect the physical and mental health of pregnant women but also cause anxiety [4], depression [5], and other symptoms of pregnant women and have a continuous impact on the growth and development of the fetus. Severe sleep problems of pregnant women can cause undesirable consequences such as premature birth [6, 7] and abortion [8] and bring heavy spiritual and economic burdens to pregnant women's families and society.

The article "Building and Realizing the Obstetrics and Gynecology Nursing Management Platform by Computer Information Technology under the Concept of Mindfulness Intervention" was retracted in 2023. Reasons: suspected computer-generated content; unreliable results or conclusions; lack of ethics approval or compliance; missing or withdrawn patient consent.

Among the traditional methods for improving pregnant women's sleep quality during pregnancy, music therapy [9] and cognitive behavioural therapy [10] have certain effects, but these intervention methods are not systematic and complete. With the development of medical technology and the transformation of modern medical models, in addition to drug treatments for psychological disorders such as anxiety and depression of pregnant women, psychological intervention methods by mindfulness have begun to be widely used in the field of health promotion. Using nondrug treatment methods such as exercise and psychotherapy, pregnant women can consciously perceive the present and then have awareness to awaken the inner self and improve their ability of self-regulation. Mindfulness intervention can effectively relieve the negative emotions of pregnant women and reduce the psychological pressure of patients using various treatment methods such as sitting in meditation, yoga, walking, and meditation. In clinical treatment, mindfulness intervention has been applied to the auxiliary treatment of chronic diseases such as insomnia, anxiety, and depression, with remarkable results.

However, the use of mindfulness intervention methods for psychological intervention treatment requires higher professionalism of the interveners. Mindfulness intervention takes a long time, and the procedure is complicated. Therefore, it is mostly in the form of face-to-face group development. This approach creates certain limitations to the application of mindfulness intervention programs. Additionally, how to grasp the effective window period of sleep quality intervention timely and effectively during pregnancy is particularly critical. The development of Internet technology provides an effective new way to solve this problem. By computer information technology, the computer network Browser/Server (B/S) architecture is constructed. After carrying out mindfulness intervention on the patient's psychological state, the system will monitor the patient's physical health indicators and mental health level data in a timely manner, until the data is analyzed and experimental conclusions are drawn. This provides a feasible plan for improving the sleep quality of pregnant women during pregnancy. Additionally, it also has important practical significance for the digital and intelligent development of the medical care management platform.

The article "Building and Realizing the Obstetrics and Gynecology Nursing Management Platform by Computer Information Technology under the Concept of Mindfulness Intervention" was retracted in 2023. Reasons: suspected computer-generated content; unreliable results or conclusions; lack of ethics approval or compliance; missing or withdrawn patient consent.

In this paper, we are going to address this issue and try to establish an obstetrics and gynecology nursing management platform used to monitor and evaluate the mental health of pregnant women. Firstly, computer information technology is adopted, and the obstetrics and gynecology nursing management system is established. Secondly, after adopting the system to intervene in the mental state of patients with mindfulness, the system timely monitors the pregnant women's physical health indicators and mental health level data. With the help of the computer data analysis system, the obstetrics and gynecology management platform is built to carry out timely mindfulness interventions for pregnant women. The established system can reach high accuracy in identifying negative emotions of pregnant women, and the accuracy can reach 89.7%.

The remaining sections of this manuscript are arranged according to the following agenda items where a brief introduction of various sections is provided.

In the subsequent section, a detailed and comprehensive review of the most relevant material from the literature is presented, whereas various issues with these approaches are identified. In this section, the proposed mechanism, which is the development of an effective nursing management system for the gynecology department, is presented along with its various sections or parts. Experimental results and observations were presented to verify various claims of the proposed scheme and how it was used to resolve the issue. Finally, concluding remarks are given as the last section of the manuscript.

## 2. Literature Review

### 2.1. Recent Research on Mindfulness Intervention Therapy

In recent years, with the advancement of medical technology, the mindfulness therapy of positive psychology has attracted widespread attention. As a psychotherapy method used in clinical treatment to relieve chronic pain of patients, mindfulness intervention can produce positive therapeutic effects on patients themselves through the self-perception and psychological adjustment of patients, combined with mindfulness yoga and various meditation methods. Parsons et al. (2017) [11] used mindfulness-based cognitive therapy and mindfulness-based decompression therapy to emphasize the importance of mindfulness practice at home and analyzed and estimated participants' typical practice completion. Research results have shown that the level of practice is positively correlated with intervention results. Navarro-Haro et al. (2019) [12] have trained on mindfulness skills in the treatment of generalized anxiety disorder in primary care. Preliminary studies have shown the effectiveness of mindfulness intervention in the treatment of generalized anxiety disorder. Querstret et al. (2020) [13] used mindfulness-based decompression and mindfulness-based cognitive therapy to systematically evaluate and meta-analyze the mental health and well-being of nonclinical samples. The results of the research have important implications for the development of the public mental health agenda. Fortuna et al. (2020) [14] developed a cognitive behavioral therapy with integrated mindfulness to analyze data results for Hispanic and Latino American immigrants suffering from comorbidities. The results of the study indicate that skills related to the intermediate results studied may help Hispanic and Latino American immigrants experience continuous exposure to adversity and traumatic stress. Pardos-Gascón et al. (2021) [15] pointed out the different effects of mindfulness therapy on chronic pain and conducted a systematic evaluation. Results show that in central sensitization syndrome, pain-related variables tend to improve with treatment. Additionally, it also proved that in all diagnoses, mindfulness intervention is superior to conventional care. Hunter-Jones et al. (2021) [16] evaluated the results of the process of mindfulness-based cognitive therapy for acquired immune deficiency syndrome (AIDS) women and showed that cis and transgender women were very satisfied with the intervention and showed improvement in symptoms of depression and stress. By collecting data on acceptability, research has shown that mindfulness-based interventions have a significant impact on treatment outcomes. Geurts et al. (2021) [17] have conducted research on mindfulness-based cognitive therapy in routine clinical practice. The study indicates that, in addition to baseline severity, specific diagnostic categories or other investigative modifiers affect treatment efficiency. Reyes (2021) [18] used mobile applications to learn the effects of mindfulness treatment through applied research, which provided a basic theoretical framework for using mindfulness intervention theory to improve treatment compliance. In summary, relevant clinical studies have been conducted on the treatment of patients by the concept of mindfulness intervention. Compared with traditional treatment methods, mindfulness intervention theory is more effective in treating patients.

The article "Building and Realizing the Obstetrics and Gynecology Nursing Management Platform by Computer Information Technology under the Concept of Mindfulness Intervention" was retracted in 2023. Reasons: suspected computer-generated content; unreliable results or conclusions; lack of ethics approval or compliance; missing or withdrawn patient consent.

### 2.2. Information Technology and Construction of Medical Care Management Platform

In the context of new health care reform, building an online medical care management platform via the Internet has become an important technical means to realize smart medical care. Cao et al. [19] (2018) have practiced and explored regional medical device management platforms via the Internet of Things (IoT). The results show that a medical device data platform by the mobile Internet can effectively reduce operating costs and improve the efficiency of device data collection. Steinhart et al. [20] (2019) used the IoT to perform patient clinical management practices. The results show that the IoT system can improve the effect of treatment evaluation. Lee et al. [21] (2020) developed and researched a personal health record management platform by blockchain technology. The built platform has become a model of a cross-regional medical data exchange management platform, which can be used for transnational precision medicine and individualized medicine. Semenov et al. [22] (2020) provided effective data support for clinical decision-making through the development of a medical data management platform, solved the problem of the convenience of obtaining clinical decision support services, and improved the service and nursing level of medical staff. Rohela et al. [23] (2021) have built a health monitoring and management platform for patients with heart disease and hypertension. The results show that the electronic health kit is an effective tool to help reduce hypertension and the potential risk of heart disease. Van Rheenen et al. [24] (2021) conducted a study on the management of children with Crohn's disease and determined that the key to early detection of high-risk patients with complex diseases is to reduce intestinal damage. This discovery can provide advanced guidance and long-term medical services for young people suffering from diseases. Chela et al. [25] (2021) reviewed the medical management of inflammatory bowel disease during the corona virus disease 2019 (COVID-19) epidemic. The results show that the use of new platforms such as telemedicine to provide clinical care can help prevent the further spread of infectious diseases.

## 3. Establishment of a Nursing Platform for Obstetrics and Gynecology

### 3.1. Platform Requirement Analysis and Overall Architecture Construction

By the latest relevant standards of medical nursing [26–28], and drawing on the most advanced comprehensive electronic case application cases, the implemented system platform will provide a structured and integrated electronic medical record system for obstetricians, gynecologists, and nurses. This achieves a high degree of sharing and utilization of electronic information. The system is used to track, record, and complete daily work in time for the daily nursing status of obstetrics and gynecology patients. It can capture patient care in medical scenarios through smart sensors, thereby reducing data redundancy and delay. Additionally, intelligent sensor interaction technology is used to collect information from obstetrics and gynecology patients in a timely manner. The data collection system is used to collect information and forward it to the medical care terminal. On this basis, the IoT is used to digitize all patient information elements of the system, and a virtual medical care service platform is reconstructed in the cyberspace. The situation of the coexistence and virtual integration of the nursing system of the physical dimension and the digital system of the information dimension has finally been formed. Therefore, physical systems and digital systems coexist and merge in the information dimension. For the detection of the patient's mental state, the system can provide historical data queries of the patient's treatment. The system will also monitor the patient's body indicators, the stability, and the scalability of data storage. The architecture of the distributed IoT nursing system that collects data by dynamic vision sensors is shown in Figure 1.

The article "Building and Realizing the Obstetrics and Gynecology Nursing Management Platform by Computer Information Technology under the Concept of Mindfulness Intervention" was retracted in 2023. Reasons: suspected computer-generated content; unreliable results or conclusions; lack of ethics approval or compliance; missing or withdrawn patient consent.

### 3.2. Patient Admission Assessment and Management Module

In the obstetrics and gynecology nursing management platform [29], the admission evaluation and management module includes functions such as admission assessment entry and admission assessment query. The nurse enters the basic information and medical history information of the patient according to the requirements of the hospital, and conducts a safety assessment of the patient's care level, and adjusts its safety care level in time. The doctor can inquire about the patient's assessment information and print out the admission assessment form. Additionally, the nurse manages the basic information of the patient and takes care of the patient according to the inquired medical order information corresponding to the patient. In the background of the system, the head nurse can formulate corresponding care plans according to the level of care set by the doctor and implement them for the patients. Nurses can view the care plans of the patients they are responsible for and implement them according to plan reminders. The management module of patient admission evaluation is shown in Figure 2.

Wireless smart sensors [30] are used to monitor the data of various vital signs of pregnant women and fetuses. The data collection sensor is mainly responsible for monitoring the physiological parameters of the fetus and the surrounding environmental conditions. The data collection sensor provides the necessary information for the computer or doctor to analyze the existing condition. After the local monitoring terminal collects and analyses the data, it sends the data to the hospital monitoring centre via the Internet. The specific process framework is shown in Figure 3.

The article "Building and Realizing the Obstetrics and Gynecology Nursing Management Platform by Computer Information Technology under the Concept of Mindfulness Intervention" was retracted in 2023. Reasons: suspected computer-generated content; unreliable results or conclusions; lack of ethics approval or compliance; missing or withdrawn patient consent.

### 3.3. Measurement of Maternal and Fetal Heart Rate by Doppler Effect

In the daily care and management of pregnant women in the Department of Obstetrics and Gynecology, the heart rate of the fetus is an important indicator. The physical and psychological conditions of pregnant women will inevitably affect the healthy development of the fetus. Ultrasound is used to monitor the frequency of emitted and received sound waves [31]. The difference between the frequencies of the emitted and received sound waves is represented by the Doppler frequency shift *f*_*D*_, and the calculation is shown as follows:

(1) $$\begin{array}{c} f_{D}=\pm 2V\times \frac{f_{0}}{C}. \end{array}$$

Among them, *f*_0_ represents the frequency of transmitting ultrasonic waves. *C* is the speed of sound. *V* is the relative speed of movement between objects. The sign indicates the direction of movement of the object. The positive sign indicates the direction close to the sound source. The negative sign indicates the direction away from the sound source.

When there is a certain angle between the direction of interface movement and the direction of ultrasound, the calculation of Doppler Shift *f*_*D*_ is shown as follows:

(2) $$\begin{array}{c} f_{D}=\pm 2V\times \cos\theta \times \frac{f_{0}}{C}. \end{array}$$

Among them, *θ* represents the angle between the direction of interface movement and the direction of ultrasonic waves. *V* × cos*θ* represents the projection of the actual operating speed in the ultrasonic direction. Let *f*(*t*) be the square integrable function. When monitoring the fetal heart rate, the signal transmission adopts the method of multiscale wavelet analysis by Fourier transform analysis. The continuous wavelet transform function of *f*(*t*) is shown as follows:

(3) $$\begin{array}{c} WT_{f}\left(a,b\right)={\left|a\right|}^{-1/2}\int_{-\infty }^{\infty }f\left(t\right)\psi \left(\frac{t-b}{a}\right)\text{d}t,\;a\neq 0. \end{array}$$

Among them, *a* is the expansion factor, and *b* is the translation factor, which is expressed in the form of an inner product as follows:

(4) $$\begin{array}{c} WT_{f}\left(a,b\right)=f,\psi_{a,b}. \end{array}$$

Among them, *ψ*_*a*,*b*_(*t*)=|*a*|^−1/2^*ψ*((*t* − *b*)/*a*).

The wavelet analysis method is used to process the fetal heart rate signal. Firstly, the order of Wavelet decomposition is determined. After the fetal heart rate signal is processed by Wavelet, the high-frequency signal and the low-frequency signal are separated. The high-frequency noise signal is directly removed after being processed, and the low-frequency signal is quickly filtered after inverse transformation processing, and then the instantaneous fetal heart rate value is calculated [32]. The process and framework of doctors and nurses' nursing operations on pregnant patients are shown in Figure 4:

The article "Building and Realizing the Obstetrics and Gynecology Nursing Management Platform by Computer Information Technology under the Concept of Mindfulness Intervention" was retracted in 2023. Reasons: suspected computer-generated content; unreliable results or conclusions; lack of ethics approval or compliance; missing or withdrawn patient consent.

### 3.4. Experimental Environment Parameter Setting

After completing the requirements analysis, the overall system architecture, and the design of each module unit, the constructed system needs to be pressure tested to ensure that the system can operate safely and stably. Since the system design has two ports, Web and APP, it is necessary to test the server, Web, and APP at the same time. Among them, the server-side operating system is Windows Server 2008. The database is using SQL Server 2008 R2 version. The hardware is 1T solid state drive and has 4G processing memory. The Web terminal uses the Windows 7 operating system, equipped with 2G processing memory and a 500G solid-state hard drive, and the browser kernel is Chrome. The APP-side experiment configuration is mainly considered from two aspects: hardware and software. In terms of software, the experimental platform is configured as a Dell computer, equipped with an Intel(R) i5-7500, 3.40 GHz, 8 GB RAM, and the Windows 10 operating system. In addition, the system is also equipped with the CUDA 9.0 + cuDNN 7.2 version of TensorFlow-GPU, the advanced packaging library Keras, and the data processing library sklearn. The algorithm programs involved are all written in the Python language. Anaconda and PyCharm are used as development platforms. The corresponding version numbers of the software tools used in the experiment are TensorFlow-GPU 1.10.0, Anaconda 3-4.1.0, and Python 3.6.

Through system testing, the treatment method of mental state mindfulness intervention for pregnant women using the obstetrics and gynecology nursing management platform is compared with traditional treatment methods. Whether the pregnant woman suffers from mental depression is judged and identified. From the perspectives of accuracy, precision, recall, and *F*1 value, the recognition accuracy of the system model is analyzed. The reliability of the improved obstetrics and gynecology nursing management platform can be verified. In addition, the data security transmission performance of the system model is evaluated. From the average transmission rate, average leakage rate, average delay, and packet loss rate of system data, the security of system network data transmission is evaluated.

## 4. Results and Evaluation

### 4.1. Evaluation of System Disease Recognition Performance Results

The concept of mindfulness intervention is adopted for psychological intervention and adjustment of negative psychological state for obstetrics and gynecology patients. The patient's disease recognition accuracy is evaluated. In order to study the detection effect of the system on obstetrics and gynecology patients under the concept of mindfulness intervention, the recognition accuracy, precision, recall rate, and F1 value of the system are compared with those of traditional methods. The results are shown in Figures 5–8. Additionally, as the number of model iterations increases, the average time delay and maximum waiting time of the system are shown in Figures 9 and 10.

The article "Building and Realizing the Obstetrics and Gynecology Nursing Management Platform by Computer Information Technology under the Concept of Mindfulness Intervention" was retracted in 2023. Reasons: suspected computer-generated content; unreliable results or conclusions; lack of ethics approval or compliance; missing or withdrawn patient consent.

In Figures 5 and 6, as time increases, the recognition accuracy and precision of the traditional method and the adopted system method will increase. If enough time is given, the final recognition accuracy and precision of the algorithm can reach the expected effect value. However, compared with traditional methods, using the proposed system for psychological intervention and mental state recognition of pregnant women, the recognition accuracy rate can reach about 90%. Compared with the traditional method, the recognition accuracy is improved by at least 7.8%. The proposed method improves the recognition accuracy by 6.5% compared with the traditional method. The highest recognition rate can reach 89.7%. The proposed method greatly improves the accuracy and accuracy of recognition.

Figures 7 and 8 show that after the system has processed the data for a certain period, the recognition recall rate of the proposed system model can reach about 75%. Compared with the 68% recognition recall rate of the traditional method, it is improved by at least 7.0%. In terms of changes in F1 value, the nursing system is used to evaluate the mental state and identify diseases of obstetrics and gynecology patients. As time goes by, the *F*1 value is getting bigger and bigger. After 120 s, the recognized *F*1 value after the intervention of the system reached 98.6%. The proposed system model greatly improves the judgment and evaluation level of pregnant women's psychological status.

For the average delay and maximum waiting time of the system, as the number of model iterations increases, the average delay time of the system using the two methods after 60 iterations is below 5 s. However, the average delay of the proposed system can be reduced to 3.4 s, which can be reduced by 1.2 s compared to the traditional method. In terms of the waiting time of the system, the maximum waiting time of the proposed system model can be reduced to about 21 s after 60 iterations, which is in sharp contrast with the 28.4 s maximum waiting time of the traditional method. The proposed system can greatly reduce the waiting time for doctors and nurses to query patient data and improve the efficiency of obstetrics and gynecology nursing management.

The article "Building and Realizing the Obstetrics and Gynecology Nursing Management Platform by Computer Information Technology under the Concept of Mindfulness Intervention" was retracted in 2023. Reasons: suspected computer-generated content; unreliable results or conclusions; lack of ethics approval or compliance; missing or withdrawn patient consent.

### 4.2. Analysis of the Security Performance of Network Data Transmission in Different Architectures of the System

From the aspects of the average delivery rate, average leakage rate, average delay, and packet loss rate of network data security transmission performance, the performance of the B/S architecture adopted by the proposed system is further compared with the performance of the traditional C/S architecture. The results are shown in Figures 11–14.

In Figure 11, the average data transmission rate of the system network using the C/S architecture is higher, and the average transmission rate has reached 90%. The average data transmission rate of the system network under the B/S architecture can only reach up to 90%.  Figure 12 shows the average data leakage rate under the two network architectures. The data transmission leakage rate under the B/S network architecture is even smaller, with an average of about 40%, which is 9.6% less than the C/S architecture. Therefore, although the selected B/S architecture has a loss in the average transmission rate, it can obtain a smaller average data leakage rate, so the performance is better.

By comparing the average data delay and data packet loss rate of different network architectures, in terms of average delay, the delay decreases as the amount of transmitted data increases. The average delay used by the proposed system is basically stable at about 340 ms, as shown in Figure 13. In the packet loss rate analysis shown in Figure 14, the system has a higher packet loss rate under the C/S architecture, and there may be hidden terminal problems and packet loss. The system model of the B/S architecture adopted by the proposed system has a low packet loss rate, which does not exceed 10%. This is because the B/S architecture system will balance the transmission data. From a different data transmission point of view, although the proposed B/S system network architecture performs poorly in terms of transmission rate, it has the characteristics of a higher average delivery rate, the lowest average leakage rate, and lower latency. The proposed system shows good network data security transmission performance.

## 5. Conclusion

Depression during pregnancy is a mental health issue that deserves attention. During pregnancy, pregnant women who have been in a state of depression and anxiety for a long time are extremely detrimental to the healthy development of the fetus. By adopting the method of mindfulness intervention to provide mental health care for obstetrics and gynecology patients, the mindfulness intervention level and acceptance level of pregnant women can be effectively improved. In clinical nursing, the obstetrics and gynecology nursing management platform is used to monitor the physical health of pregnant women in a timely manner to help pregnant women cope with their negative emotions during pregnancy. The results show that the established system can achieve 90% accuracy in identifying negative emotions of pregnant women, and the accuracy can reach 89.7%. The established system can timely and accurately intervene and regulate the pregnant woman's unhealthy mental state. This has important application value for the mental health control of pregnant women during pregnancy. However, some shortcomings are unavoidable, which are as follows: (i) The lack of blood indicator monitoring for the evaluation of depression and anxiety during pregnancy may lead to unavoidable subjective errors of the subject. (ii) The positive effect of mindfulness intervention may be related to the attention of medical staff, which was unable to determine the effective degree of intervention in the experiment. In the future, in order to achieve better clinical trial results, multicentre, large-sample data research will be carried out. Moreover, the proposed system can be further extended by considering other departments of the hospitals such as the intensive care unit and other relevant departments or wards.

The article "Building and Realizing the Obstetrics and Gynecology Nursing Management Platform by Computer Information Technology under the Concept of Mindfulness Intervention" was retracted in 2023. Reasons: suspected computer-generated content; unreliable results or conclusions; lack of ethics approval or compliance; missing or withdrawn patient consent.

## Figures and Tables

**Figure 1:** System architecture diagram of the distributed IoT nursing system.

**Figure 2:** Sample diagram of the patient admission management system module.

**Figure 3:** Data collection and management of the maternal care system.

**Figure 4:** Flow chart of doctors and nurses caring for pregnant women.

**Figure 5:** The curve of recognition accuracy of system with time.

**Figure 6:** The curve of recognition accuracy varying with time.

**Figure 7:** The system's identification recall rate versus time curve.

**Figure 8:** The system's identification *F*1 value change curve diagram over time.

**Figure 9:** The average time delay of the system as the number of model iterations increases.

**Figure 10:** The maximum waiting time of the system as the number of model iterations increases.

**Figure 11:** Comparison of the average data transmission rate under different network architectures.

**Figure 12:** Comparison of the average data leakage rate of the system under different network architectures.

**Figure 13:** Comparison of the average data delay of the system under different network architectures.

**Figure 14:** Comparison of system data packet loss rates under different network architectures.

The article "Building and Realizing the Obstetrics and Gynecology Nursing Management Platform by Computer Information Technology under the Concept of Mindfulness Intervention" was retracted in 2023. Reasons: suspected computer-generated content; unreliable results or conclusions; lack of ethics approval or compliance; missing or withdrawn patient consent.

## Data Availability

The datasets used and/or analyzed during the current study are available from the corresponding author upon reasonable request.
